RETRACTED

# Breast cancer surgery in elderly patients: postoperative complications and survival

**DOI:** 10.1186/1471-2482-13-S2-S25

**Published:** 2013-10-08

**Authors:** Nicola Rocco, Corrado Rispoli, Gennaro Pagano, Giuseppe Rengo, Rita Compagna, Michele Danzi, Antonello Accurso, Bruno Amato

**Affiliations:** 1 Department of Biomedical, Surgical and Dental Sciences, University of Milan, Milan, Italy; 2 Department of General Surgery, Cardinale Ascalesi Hospital - ASL NA1, Naples, Italy; 3 Dept. of Translational Medical Sciences, University "Federico II" of Naples, Naples, Italy; 4 Department of General, Geriatric, Oncologic Surgery and Advanced Technologies, University "Federico II" of Naples, Naples, Italy

## Abstract

**Aims and background:**

Old age is associated with comorbidity and decreased functioning which influences treatment decisions in elderly breast cancer patients. The purpose of this study was to identify risk factors for complications after breast cancer surgery in elderly patients, and to assess mortality in patients with postoperative complications.

**Methods:**

We retrospectively considered all female patients aged 65 years and older with invasive and in situ breast cancer who were diagnosed and treated between 1997 and 2012 in the Department of General and Geriatric Surgery of the University of Naples "Federico II".

**Results and conclusion:**

449 patients received surgery, of whom 18,2% (n = 82) developed one or more postoperative complications. The odds ratio of having postoperative complications show an increase with age, reaching statistical significance only for patients older than 85 [OR 5,75 (95% confidence interval 2,38-14,04); p < 0,001]. Number of concomitant diseases [OR 2,51 (95% CI 1,17 - 5,45); p = 0,01 for 3 or more concomitant diseases] and polypharmacy [OR 16,7 (95% CI 9,12 - 30,58); p < 0,0001) are associated to an increased risk of postoperative complications. Overall survival was worse in patients with postoperative complications [HR 2,06 (95% CI 1,52-2,70), p < 0,001]. This increased risk of mortality is probably due to geriatric parameters such as comorbidity or poor physical function, more than to higher complication rates.

## Introduction

In developed countries, 40% of breast cancer patients are older than 65 years of age at diagnosis and this percentage is increasing [1]. Old age is predictive for comorbidity and decreased functioning [2,3]. Therefore, these factors might influence treatment decisions in elderly breast cancer patients. Previous studies have shown that elderly breast cancer patients receive less aggressive treatment [4] and have a higher disease-specific mortality, even with 65% of breast cancer patients above 75 years dying from other causes than breast cancer [5].

RETRACTED

The most recent guidelines of the International Society of Geriatric Oncology and the European Society of Breast Cancer Specialists (EUSOMA) advise breast conserving surgery with whole-breast radiotherapy or mastectomy followed by postoperative radiotherapy in selected patients as standard care for elderly breast cancer patients [6]. However, the National Comprehensive Cancer Network guidelines state that omission of radiotherapy may be considered in patients of 70 years or older with stage I estrogen receptor-positive breast cancer who undergo a lumpectomy with negative margins and are receiving endocrine therapy [7]. This shows that there is still no consensus on how to treat elderly breast cancer patients. Also, elderly patients are often not treated according to guidelines [8,9]. Comorbid conditions and frailty are, besides age and patient and physician's preference, important reasons to deviate from the guidelines [10,11]. Besides, treatment strategies for elderly breast cancer patients are mostly not evidence-based because elderly are often not included in clinical trials due to age restrictions or comorbidity [12].

Breast surgery is generally considered as low-morbidity surgery [13]. However, a variety of complications can occur with serious consequences. For example, surgical site infections can lead to increased morbidity, additional costs and delay of postoperative adjuvant therapies [13].

In order to develop evidence-based guidelines for tailored care of breast cancer in the elderly, it is important to investigate the occurrence of complications of surgery in this specific group. Only few studies concerning postoperative complications in elderly breast cancer patients have been performed, often with a limited number of patients [11,14,15]. Therefore, the objective of this study was to identify risk factors for postoperative complications in elderly breast cancer patients, and to evaluate overall survival in patients with postoperative complications compared with patients without postoperative complications.

## Methods

We considered all consecutive female patients aged 65 years and older with invasive and in situ breast cancer who were diagnosed and treated between 1997 and 2012 in the Department of General and Geriatric Surgery of the University of Naples "Federico II".

We reviewed the charts of these patients and collected information on specific treatments, comorbidities, adverse events, geriatric parameters, body mass index (BMI), smoking and mortality.

For this study, all patients with breast cancer stage I-IV and in situ of all histological subtypes who were treated with breast conserving surgery or mastectomy were included. If patients received breast-conserving surgery (BCS) followed by mastectomy, the most extensive surgery was used for analyses. Stage was described using the pathological tumor-node-metastasis (TNM) classification, as valid in the year of diagnosis. If the pathological stage was missing, clinical stage was used. Axillary surgery was defined as a sentinel node procedure or an axillary lymph node dissection. Again, the most extensive axillary surgery was used for the analyses.

RETRACTED

To compare different age groups, patients were categorized into five groups: 65-69, 70-74, 75-79, 80-84, and 85 years or older.

Number of concomitant diseases was categorized in four groups: no concomitant disease, 1 concomitant disease, 2 concomitant diseases and 3 or more concomitant diseases [16]. BMI was analyzed in three groups: <20, 20-25, and >25.

In case of missing data, patients were not excluded from the analyses, but analyzed in a separate group (unknown).

The possible postoperative complications were wound infections (including abscesses), bleeding, hematoma, seroma, anemia, cardiovascular complications, thrombo-embolisms and other complications. The primary outcome was defined as having one or more of these complications.

## Statistical analyses

All statistical analyses were two-sided. A p value smaller than 0.05 was considered as significant.

The following risk factors for having at least one post-operative complication were assessed in univariable logistic regression models: age (in groups per 5 years), stage according to the TNM-classification, most extensive surgery, most extensive axillary surgery, number of comorbid conditions, polypharmacy (5 or more types of drugs per day), neoadjuvant treatment, BMI, and smoking at time of surgery.

## Results

### Patient characteristics

Overall, 449 patients of 65 years and older with invasive and in situ breast cancer underwent BCS or mastectomy and were included for analyses. Patient characteristics are shown in Table 1.

**Table 1:** Patients characteristics.

PATIENTS' CHARACTERISTICS	n (449)	%
MEDIAN AGE (range)	76.0 (65-92)	

AGE		

65-69	131	29,5%

70-74	114	25,1%

75-79	87	19,3%

80-84	68	15,2%

>85	49	10,9%

N OF CONCOMITANT DISEASE		

0	113	25,2%

1	112	25,0%

2	106	23,6%

> = 3	118	26,2%

TNM STAGE		

IN SITU	17	3,9%

I	168	37,5%

II	180	40,1%

III	39	8,8%

IV	4	1,0%

UNKNOWN	41	8,7%

NEOADJUVANT TREATMENT		

NO NEOADJUVANT TREATMENT	436	97%

NEOADJUVANT CHEMOTHERAPY	13	3%

BREAST SURGERY		

BREAST CONSERVING SURGERY	125	28%

MASTECTOMY	324	72%

AXILLARY SURGERY		

NO AXILLARY SURGERY	40	9%

SENTINEL NODE BIOPSY	180	40%

AXILLARY LYMPH NODE DISSECTION	229	51%

BMI		

<20	4	1%

20-25	86	19,1%

>25	135	30,1%

UNKNOWN	224	49,8%

POLYPHARMACY		

NO	354	79%

YES	95	21%

SMOKING AT TIME OF DIAGNOSIS		

NO	276	61,5%

YES	31	6,9%

UNKNOWN	142	31,6%

Most patients (72%) were treated with mastectomy. The majority of patients (74.8%) had at least one concomitant disease. Few patients (3.0%) received neoadjuvant treatment. 21% of the patients used 5 or more types of drugs per day. BMI values were missing in 224 patients (49.8%) and data about smoking were missing in 142 patients (31.6%). Median follow up was 7.5 years (range 0.01 -15.0).

RETRACTED

### Postoperative complications

Overall, 18.2% of patients developed 1 or more postoperative complications (Table 2). The most frequent complications were seroma (n = 21) and wound infection (n = 17).

**Table 2:** Complications in different age groups.

	TOTAL	65-69	70-74	75-79	80-84	> = 85
ALL COMPLICATIONS	82 (18,2%)	13 (9,9%)	15 (13,2%)	17 (19,5%)	18 (26,5%)	19 (38,8%)

WOUND INFECTION	17 (3,8%)	3	4	4	3	3

BLEEDING	14 (3,2%)	4	2	2	3	3

HEMATOMA	14 (3,2%)	3	2	4	3	2

SEROMA	21 (4,8%)	2	4	5	4	6

ANEMIA	2 (0,4%)	0	0	0	1	1

CARDIOVASCULAR COMPLICATION	8 (1,4%)	0	2	2	2	2

THROMBO-EMBOLISM	4 (1,0%)	1	1	0	1	1

OTHER COMPLICATIONS	2 (0,4%)	0	0	0	1	1

As shown in Table 3, the odds ratio (OR) for developing a postoperative complication increased with age (OR for patients aged > 85 years was 5.75 (95% confidence interval 2.38-14.04, p < 0.001) in a univariable logistic regression model).

**Table 3:** Association between patient, tumor characteristics, treatment and occurrence of postoperative complications.

	N OF PATIENTS WITH COMPLICATION (%)	OR	95% CI	p value
AGE				

65-69	13 (9,9%)	Ref		

70-74	15 (13,2%)	1,37	0,58-3,24	ns

75-79	17 (19,5%)	2,20	0,95-5,16	ns

80-84	18 (26,5%)	3,27	1,40-7,72	0,004

> = 85	19 (38,8%)	5,75	2,38-14,04	<0,001

N OF CONCOMITANT DISEASE				

0	13 (12,0%)	Ref		

1	20 (18,3%)	1,67	0,74-3,80	ns

2	20 (18,5%)	1,79	0,80-4,07	ns

> = 3	29 (24,6%)	2,51	1,17-5,45	0,01

POLYPHARMACY				

NO	27 (7,6%)	Ref		

YES	55 (57,9%)	16,65	9,12-30,58	<0.0001

BREAST SURGERY				

BREAST CONSERVING SURGERY	29 (23,2%)	Ref		

MASTECTOMY	53 (16,4%)	0.65	0,38-1,11	ns

AXILLARY SURGERY				

NO AXILLARY SURGERY	5 (12,5%)	Ref		

SENTINEL NODE BIOPSY	31 (17,2%)	1,46	0,49-4.60	ns

AXILLARY LYMPH NODE DISSECTION	46 (20,1%)	1,76	0,61-5,43	ns

NEOADJUVANT CHEMOTHERAPY				

NO NEOADJUVANT TREATMENT	76 (17,4%)	Ref		

NEOADJUVANT CHEMOTHERAPY	6 (46,1%)	4,06	1,17-13,92	<0,05

TNM STAGE				

IN SITU	4 (23,5%)			

I	27 (16,1%)	Ref		

II	25 (13,9%)	0,84	0,45-1,58	ns

III	8 (20,5%)	1,35	0,51-3,49	ns

IV	1 (25%)	1,74	0,07-19,99	ns

UNKNOWN	17 (41,5%)			

BMI				

<20	1 (25%)	2,06	0,08-25,85	ns

20-25	12 (14%)	Ref		

>25	31 (23%)	1,84	0,84-4,08	ns

UNKNOWN	38 (17%)			

SMOKING AT TIME OF DIAGNOSIS				

NO	46 (16,7%)	Ref		

YES	11 (35,5%)	2,75	1,14-6,54	<0,05

UNKNOWN	25 (17,6%)			

A higher number of concomitant diseases was associated with a higher risk of postoperative complications (patients without concomitant disease functioned as a reference; OR was 1.67 (95% CI 0.74-3.80), 1.79 (95% CI 0.80-4.07) and 2.51 (95% CI 1.17-5.45; p = 0.01) in patients with 1, 2 and 3 or more concomitant diseases, respectively).

RETRACTED

Similarly, polypharmacy was strongly associated with risk of complications (OR 16.7 (95% CI 9.12-30.58), p < 0.0001).

Furthermore, patients who received a mastectomy and patients who underwent axillary lymph node dissection had more complications than patients who were treated with breast conserving surgery and less extensive axillary surgery.

Smoking increased the odds for developing a complication with an OR of 2.75 (95% CI 1.14-6.54, p < 0.05).

There was no significant association between BMI and postoperative complications.

Overall survival was worse in patients with postoperative complications [HR 2,06 (95% CI 1,52-2,70), p < 0,001] (Table 4). This increased risk of mortality is probably due to geriatric parameters such as comorbidity or poor physical function, more than to higher complication rates.

**Table 4:** Survival analyses for one or more postoperative complications versus no postoperative complications.

	DEATHS	5-YEAR SURVIVAL (%)	HR	95% CI	p value
OVERALL SURVIVAL	133	70			

No postoperative complications	91	75	Ref		

Postoperative complications	42	49	2,06	1,52-2,70	< 0,001

## Discussion

This study shows that the number of concomitant diseases and polypharmacy are strongly related to the occurrence of postoperative complications in elderly breast cancer patients.

Patients treated with mastectomy had more complications than patients who received breast conserving surgery.

Elderly patients had complications more often, but after adjustment for tumor stage, comorbidity, and treatment, only a trend for increasing risk of complications in higher age groups was observed.

Overall survival was worse in patients with one or more postoperative complications.

The increased risk for early and late overall mortality is probably not due to the complications in itself, but can be explained by the frail state of the patients who develop postoperative complications, since comorbidity in itself increases the risk of mortality in elderly breast cancer patients [17,18].

Concerning the impact of comorbidity on developing postoperative complications, Houterman et al. [15] concluded from an observational study that comorbidity and age did not influence the occurrence of complications after treatment. The study included only 154 patients aged 70 years or older, and investigated complications of all types of therapy in the first year after diagnosis. Also, patients who did not receive surgery were included in this study. Therefore, this study differs considerably from the current study, which might explain the differences in outcome. Another study by Janssen-Heijnen et al. [14] also found no association between comorbidity and postoperative complications. Again, this study included only 490 patients with breast cancer, of whom only 192 were older than 65. Since the impact of comorbid disease is the highest in the eldest elderly, this might explain the differences with the current study.

RETRACTED

A recent Danish study [19] found that older age and mastectomy increases the risk of re-operation due to bleeding in breast cancer surgery. These results were confirmed in the current study.

Another study [20] found that BMI > 25, diabetes, and smoking were predictors of wound complications. In the current study, BMI was not related to risk of postoperative complications, which might be explained by missing values in about 50% of patients, since BMI registration in a chart may not be missing at random.

Since elderly patients are rarely included in clinical trials [12], large cohort studies are of great importance in this population. These studies are a good way of studying complications of treatment, since data are unbiased and the studies generally contain more patients [21].

This study also has some limitations. Due to the retrospectively collection of data, there might have been an underestimation of the number of complications. However, in these data, 18.2% of patients developed at least one complication, and this is even higher than a recent study in a large cohort in the U.S. [20] which reported a 30-day morbidity rate for all breast cancer procedures of 5.6%. The most common complications were wound infections. Therefore, these data seem to accurately reflect general practice and correspond with previous studies.

A meta-analysis has confirmed that hormonal treatment as monotherapy is inferior to surgery (with or without hormonal treatment) for the local control and progression-free survival of breast cancer in medically fit older women [22-25].

However, in Italy, elderly patients receive less surgery and more hormonal therapy as monotherapy than younger patients, even in lower stages of disease [4].

This suggests that patients might be undertreated due to fear of morbidity and mortality in breast cancer surgery. Although elderly patients with comorbidity do have a higher risk of postoperative complications, relative mortality was not higher in this group and therefore suggests that omitting surgery because of fear for treatment-related mortality is only justified in vulnerable elderly patients. The question remains how to identify this specific group. Therefore, future prospective studies are needed to identify patients at risk for postoperative complications, and to develop tailored care for elderly breast cancer patients.

RETRACTED

## List of abbreviations

BMI: body mass index

## Competing interests

The authors declare that they have no competing interests.

## Authors' contributions

N.R, C.R: conception and design, interpretration of data, given final approval of the version to be published.

G.P, G.R, R.C, M.D: acquisition of data, drafting the manuscript, given final approval of the version to be published

A.A, B.A: critical revision, interpretation of data, given final approval of the version to be published

## Authors' information

NR: PhD in Thoracic Surgery at University of Milan.

CR: Specialist in General Surgery, Cardinale Ascalesi Hospital of Naples.

GP: Resident in Geriatrics at University Federico II of Naples.

GR: Resident in Cardiology at University Federico II of Naples.

R.C.: doctoral fellow in Surgery at University Federico II Naples.

MD: Aggregate Professor of Surgery at University "Federico II" of Naples.

AA: Specialist in General Surgery, University Federico II of Naples.

BA: Associate Professor of Surgery at University "Federico II" of Naples.

## Declarations

Publication of this article has come from personal funds.

This article has been published as part of *BMC Surgery *Volume 13 Supplement 2, 2013: Proceedings from the 26th National Congress of the Italian Society of Geriatric Surgery. The full contents of the supplement are available online at http://www.biomedcentral.com/bmcsurg/supplements/13/S2.
